# Effect of Salinity on Biomass Yield and Physiological and Stem-Root Anatomical Characteristics of Purslane (*Portulaca oleracea* L.) Accessions

This article has been retracted.

**DOI:** 10.1155/2015/105695

**Published:** 2015-02-23

**Authors:** Md. Amirul Alam, Abdul Shukor Juraimi, M. Y. Rafii, Azizah Abdul Hamid

**Affiliations:** ^1^Department of Crop Science, Faculty of Agriculture, Universiti Putra Malaysia (UPM), 43400 Serdang, Selangor, Malaysia; ^2^Institute of Tropical Agriculture, Universiti Putra Malaysia (UPM), 43400 Serdang, Selangor, Malaysia; ^3^Faculty of Food Science and Technology, Universiti Putra Malaysia (UPM), 43400 Serdang, Selangor, Malaysia

## Abstract

13 selected purslane accessions were subjected to five salinity levels 0, 8, 16, 24, and 32 dS m^−1^. Salinity effect was evaluated on the basis of biomass yield reduction, physiological attributes, and stem-root anatomical changes. Aggravated salinity stress caused significant (*P* < 0.05) reduction in all measured parameters and the highest salinity showed more detrimental effect compared to control as well as lower salinity levels. The fresh and dry matter production was found to increase in Ac1, Ac9, and Ac13 from lower to higher salinity levels but others were badly affected. Considering salinity effect on purslane physiology, increase in chlorophyll content was seen in Ac2, Ac4, Ac6, and Ac8 at 16 dS m^−1^ salinity, whereas Ac4, Ac9, and Ac12 showed increased photosynthesis at the same salinity levels compared to control. Anatomically, stem cortical tissues of Ac5, Ac9, and Ac12 were unaffected at control and 8 dS m^−1^ salinity but root cortical tissues did not show any significant damage except a bit enlargement in Ac12 and Ac13. A dendrogram was constructed by UPGMA based on biomass yield and physiological traits where all 13 accessions were grouped into 5 clusters proving greater diversity among them. The 3-dimensional principal component analysis (PCA) has also confirmed the output of grouping from cluster analysis. Overall, salinity stressed among all 13 purslane accessions considering biomass production, physiological growth, and anatomical development Ac9 was the best salt-tolerant purslane accession and Ac13 was the most affected accession.

## 1. Introduction

Salinity is possibly the most imperative ecological restriction that causes extensive crop yield losses all over the world, and its threat is escalating day by day [1]. Increasing salinity reduces the average yield of major crops by more than 50% [2], and these losses are of great concern mainly for the agriculture based countries. Soil contains soluble salts of multifarious nature. High concentrations of salt impose both osmotic and ionic stresses on the plants which lead to several morphological and physiological changes [3]. A clear stunting of plants is noticed due to salinity stress [4]. Parida and Das [5] reported that the detrimental effects of high salinity on plants can be observed at the whole-plant level as the death of plants and/or decreases in productivity. High salt content, especially chloride and sodium sulphates, affects plant growth by modifying their morphological, anatomical [6], and physiological traits [7]. It is evident that there are big changes in morphology and anatomy of plants growing in saline soils [8]. Physiological responses to salinity include growth suppression and lowered osmotic potential [9]. Many researchers reported that with an increase in salinity there was a decrease in the development of the xylem. Pimmongkol et al. [10] stated that the width of vascular bundles and diameters of rice stems decreased in NaCl medium.

Many plants develop mechanisms either to exclude salt from their cells or to tolerate its presence within the cells. During the onset and development of salt stress within a plant, all the major processes such as photosynthesis, protein synthesis, and energy and lipid metabolism are affected. The earliest response is a reduction in the rate of leaf surface expansion, followed by a cessation of expansion as the stress intensifies [5]. Munns and Tester [11] stated that salt-sensitive plants have reduced survival, growth, and development when exposed to even low to moderate salinities, whereas salt-tolerant species are able to grow and reproduce even at oceanic salinities. The only way to control the salinization process and to maintain the sustainability of landscape and agricultural fields is to combat the salinization problems by environmentally safe and clean techniques, as follows: use of salt-tolerant species [12, 13].

Purslane (*Portulaca oleracea* L.) is the eighth most common plant distributed throughout the world, being a heat and drought tolerant important vegetable crop [14]. It is eaten fresh, cooked, or dried and interest in cultivating it as a food crop has increased all over the world in recent years since its identification as a rich source of *ω*3 polyunsaturated fatty acids and antioxidants [15, 16]. Moreover, purslane is promising for providing both novel biologically active substances and essential compounds for human nutrition [17]. Purslane has been proved to be more salt-tolerant than any other vegetable crops [18, 19] and can produce enough biomass under moderate salinity stress in which other vegetable crops cannot [20]. Salt-tolerant crop varieties are becoming essential in many areas of the world including Malaysia because of salt accumulation on soil, restrictions on groundwater use, and saltwater intrusion into groundwater [21]. Salt-tolerant plants have the ability to minimize these detrimental effects by producing a series of morphological, physiological, and biochemical processes [22]. It is important to understand the mechanism of physiological adaptation as well as changes in anatomical structure under salinity that may help a plant breeder to evolve a salt-tolerant variety. The present investigation was, therefore, undertaken to study the effect of salinity on biomass yield and physiological and stem-root anatomical structure of purslane.

## 2. Materials and Methods

### 2.1. Purslane Accessions and Study Location

There are about 7 types of purslane available in Malaysia [23]. In our study 13 different purslane accessions were collected from varied locations of Western Peninsular Malaysia [24]. Among those, 11 were ornamental purslane (Ac1–Ac11) and two were common purslane (Ac12 and Ac13). The experiment was conducted in a glasshouse Field-2 at the Faculty of Agriculture, University Putra Malaysia (UPM), during July to October 2013 and all chemical analyses were done at the Plant Physiology and Analytic Lab, Department of Crop Science, Faculty of Agriculture, UPM, Malaysia, and histological study was done at the Botany Laboratory in the same department.

### 2.2. Planting and Cultural Practices

Seedlings of the two common purslane accessions and cuttings of the 11 ornamental purslane accessions (as ornamental purslane does not produce seed) were first grown in plastic trays filled with rice field top soils (38.96% sand, 11.05% silt, and 49.88% clay) with pH 4.8, 2.64% organic carbon, 1.25 g cc^−1^ bulk density, and CEC of 7.06 meq 100 g^−1^ soil. Soil nutrient status was 0.17% total N, 5.67 ppm available P, 15.6 ppm available K, 3357 ppm Ca, and 319 ppm Mg. Soil water retention was 30.72% (wet basis) and 46.17% (dry basis) at field capacity. The soil belonged to the Serdang series.

Ten-day-old five seedlings or cuttings for each accession were transplanted in plastic pots (24 × 22 × 20 cm) filled with the same rice field top soil mentioned above. The plants were allowed to recover from transplanting shock and for full establishment for 29 days. During this time, plants were irrigated with tap water as and when necessary. No fertilizer was used. Five levels of salinity (0, 8.0, 16.0, 24.0, and 32.0 dS m^−1^) were used in this study which were prepared using NaCl (Merck, Darmstadt, Germany) and distilled water. Salt treatment was initiated according to the treatments 30 days after transplanting (DAT) and continued till the end of the study. In each pot, 200 mL of saline water was applied on alternate days according to the treatment. The control plants received 200 mL of distilled water. The experiment was organized in a two-factor (purslane accessions × salinity) factorial randomized complete block design with three replications. Whole plants were harvested at the ground level at 60 days after transplanting. The plants were washed under tap water and kept in cool dry place for 3 days and fresh weights were recorded. After that samples were transferred in oven and left for 3 days at 40°C to avoid sudden heat burning. Finally oven temperature was balanced at 50°C and left until proper drying. Dry weights of the whole plants for each treatment and replication were recorded before grinding.

### 2.3. Data Collection and Analysis

#### 2.3.1. Biomass Yield Data Collection

*(1) Fresh Weight.* Purslane is a very succulent plant and produces considerable amount of fresh biomass. The above ground young and fresh whole portion is edible as fresh vegetable or salad. High salinity stress causes detrimental effect on fresh biomass production of purslane limiting overall growth, plant height, number of leaves, leaf area, stem diameter, and so on. The sixty-day-old harvested fresh and surface moisture-free purslane plants were weighed in g using electric balance and mean fresh weight (FW) was calculated. The reduction of fresh biomass with reduction percentage due to salinity stress was also measured using the above formula. 

*(2) Dry Weight*. Purslane produces substantial amount of fresh biomass but due to high water contents (≥90%) dry matter production is very low. Significant amount of dry matter production is a very important criterion for any stress tolerant crop species. For initial drying just after harvesting the fresh and properly cleaned purslane samples (except root) were stored in a cool dry place for 3 days, then kept in oven at 40°C temperature for 3 days (to make them dry while being prevented from sudden burning injury), and then transferred to 70°C for another 72 hours to get constant weight. The mean dry weights (DW) were then calculated from this oven-dried sample. The dry matter reduction with percentages due to salinity stress over control was measured using the following formula:

(1) %  dry  matter  reduction=Control  treatment  value−Salinized  treatment  valueControl  treatment  value ×100.

#### 2.3.2. Physiological/Gas Exchange Data Collection

*(1) Relative Chlorophyll Content.* Chlorophyll measurements were taken with a Minolta SPAD-502 chlorophyll meter (Minolta, Japan). The chlorophyll meter (or SPAD meter) is a simple, portable diagnostic tool that measures the greenness or relative chlorophyll content of leaves. Compared with the traditional destructive methods of chlorophyll extraction, the use of this equipment saves time, space, and resources. Five leaf SPAD readings from each plant were taken and then averaged to have mean SPAD reading for each replicate. The NaCl-induced effects on total chlorophyll content were calculated comparing with the untreated control treatment value.

*(2) Net Photosynthesis Rate.* The net photosynthesis rate (*μ*mol CO_2_/m^2^/sec) from each purslane plant of a pot was determined by LI-COR, LI 6400 Portable Photosynthesis System, LI-COR, Inc., Lincoln, NE, USA, and averaged them to have the mean net photosynthetic rate. The increase or decrease in the net photosynthesis rate by the effect of different salinity levels over control plants was estimated using the same machine. 

*(3) Transpiration Rate.* The average transpiration rate (mol/m^2^/sec) of purslane plants was determined by LI-COR Portable Photosynthesis System (LI-COR, Inc., Lincoln, NE, USA). NaCl-induced changes in transpiration rate were calculated comparing with untreated control plants. 

*(4) Stomatal Conductance.* Average stomatal conductance (cm/sec) of purslane leaf was measured using LI-COR, Portable Photosynthesis System (LI-COR-6400, Inc., Lincoln, NE, USA), and the changes in stomatal conductance due to salinity stress were determined comparing with untreated control plants.

#### 2.3.3. Study of Stems and Root Histology Using Scanning Electron Microscopy

Stem and root histology of purslane plants were observed using a Scanning Electron Microscope (SEM) (JEOL JSM-5610LV, Japan). The 60-day-old purslane plants treated with five different salinity levels were pulled out carefully from the soil and washed using running tape water. The properly cleaned purslane samples were then kept in shade for 30 minutes to remove the surface moisture. The main stem and tap root were cut to lengths of 5 mm with a sharp blade. The excised stems and roots were placed in formalin acetic acid (FAA) and vacuumed for 1 hour at 650 mmHg. Specimens were postfixed in 1% osmium tetroxide for 2 hours, dehydrated for 30 minutes in each graded ethanol series of 30, 50, 70, 90, 95, and 100%, and dried in Bal-Tec CPD 030 critical point dryer apparatus. The tissues were mounted on stubs, coated with gold using Auto Fine Coater (JEOL JFC-1600, Japan) for 20 min, and viewed under Scanning Electron Microscope (JEOL JSM-5610LV, Japan).

### 2.4. Statistical Analysis

All recorded data were subjected to analysis of variance using the SAS statistical software package version 9.3 [25]. Significant differences among means were calculated using Fisher's protected least significant difference (LSD) test at 5% level of significance. Pearson's correlation coefficients (*P* ≤ 0.05) were used to draw inferences on relationships among various traits.

## 3. Results

### 3.1. Purslane Biomass Yield Analysis

#### 3.1.1. Fresh Weight

Very high significant (*P* < 0.0001) variation was observed for fresh weights in untreated control 13 purslane accessions. The highest fresh weight (341.03 g) recorded in Ac8 is an ornamental purslane and the lowest (103.67 g) found in Ac13 is a common purslane (Table 1). Fresh weights of different levels of salinity stressed purslane accessions were also affected significantly with the highest (378.15 g) in Ac9 at 24 dS m^−1^ salinity and the lowest (86.98 g) in Ac12 at 32 dS m^−1^ salinity compared to control (Table 1). The increase in fresh weight with the increasing of salinity levels was recorded in Ac1 and 8 dS m^−1^ salinity, in Ac9 at 16, 24, and 32 dS m^−1^ salinity, and in Ac13 at 8 and 16 dS m^−1^ salinity levels in comparison with untreated controls (Table 1). At 8 dS m^−1^ salinity levels fresh weight reduction was varied between 1 and 37% with the lowest reduction (0.89%) in Ac3 and the highest (36.42%) reduction in Ac8. On the other hand, 3–43%, 2–48%, and 4–55% fresh weight redactions were recorded in 16 dS m^−1^, 24 dS m^−1^, and 32 dS m^−1^ salinity, respectively. On average over all accessions, 14.36, 18.88, 21.02, and 26.09% reductions in fresh weight were noted correspondingly at 8, 16, 24, and 32 dS m^−1^ salinity, which were statistically significant (*P* < 0.05, Table 1).

#### 3.1.2. Dry Weight

Dry matter (DM) contents in untreated control plants greatly varied (*P* < 0.0001) among the 13 purslane accessions and ranged between 7.94 and 20.67 g/pot with the highest DM content in Ac6 and the lowest in Ac5 (Table 2). The dry matter contents in Ac2, Ac4, Ac8, and Ac9 were recorded as 15.39 g, 15.55 g, 16.63 g, and 15.5 g, respectively, which were statistically similar or not significant (Table 2). Nonsignificant similar results were also observed in Ac12 and Ac13. Dry matter contents were also significantly reduced by NaCl-induced salinity stress in all 13 purslane accessions with the increasing of salinity levels except Ac1 at 8 dS m^−1^ salinity, Ac9 at 16 dS m^−1^, 24 dS m^−1^, and 32 dS m^−1^, and Ac12 and Ac13 at 8 dS m^−1^ salinity where significant increasing of dry matter content was recorded (Table 2). On the other hand, the highest dry matter reduction (63.47%) was found in Ac6 at 32 dS m^−1^ salinity and the lowest reduction (1.64%) was noted in Ac5 at 24 dS m^−1^ salinity whereas the highest increase (54.19%) in dry matter content was recorded in Ac9 at 24 dS m^−1^ salinity following the lowest increase (1.83%) in Ac13 at 8 dS m^−1^ salinity (Table 2). The mean values of all the accessions revealed 11.24%, 20.91%, 23.05%, and 32.88% reductions in dry matter content, respectively, at 8 dS m^−1^, 16 dS m^−1^, 24 dS m^−1^, and 32 dS m^−1^ salinity, which were statistically significant (*P* < 0.0001, Table 2).

### 3.2. Purslane Physiological Traits Analysis

#### 3.2.1. Total Chlorophyll Content

Among all 13 purslane accessions total chlorophyll contents in untreated control plants were greatly significant (*P* < 0.0001) and ranged from 25.2 to 38.74 SPAD value; the highest chlorophyll content was recorded in Ac9 and the lowest was recorded both in Ac1 and in Ac5 (Figure 1). Chlorophyll contents in Ac3, Ac4, and Ac8 were found at 33.3, 33.4, and 33.0 SPAD value, respectively, which was not statistically significant. Chlorophyll contents in salt treated 13 purslane accessions were also reduced consequently with the increasing of salinity levels. In contrast, a bit increase in chlorophyll contents was also noted in Ac2 at 8 and 16 dS m^−1^, in Ac4 and Ac6 at 16 dS m^−1^, and in Ac8 at 8 and 16 dS m^−1^ salinity stress (Figure 1). The overall highest reduction (39.44%) in chlorophyll contents was observed in Ac7 at the highest levels 32 dS m^−1^ salinity with the lowest reduction (0.32%) in Ac11 at 8 dS m^−1^ salinity, while the highest increase (3.64%) in chlorophyll contents was found in Ac8 at 8 dS m^−1^ salinity with the lowest increase (1.82%) in the same accessions at 16 dS m^−1^ salinity levels (Table 3). On average over all accessions, 2.59% reduction, 1.17% increase, 11.21% reduction, and 18.79% reduction in total chlorophyll contents were recorded correspondingly at 8, 16, 24, and 32 dS m^−1^ salinity, which were statistically significant (*P* < 0.05, Table 3).

#### 3.2.2. Net Photosynthesis Rate

Net photosynthesis rate in untreated control plants greatly varied (*P* < 0.0001) among the 13 purslane accessions and ranged between 19.55 and 22.29 *μ*mol CO_2_/m^2^/sec with the highest photosynthesis rate in Ac2 and the lowest in Ac6 (Figure 2). Statistically similar and nonsignificant variations in net photosynthesis rate were observed in several accessions like Ac1, Ac3, Ac5, Ac10, Ac11, and Ac13 with the values 22.29, 21.89, 21.88, 21.87, 21.89, and 21.89 *μ*mol CO_2_/m^2^/sec (Figure 2). Both the negative and positive effects of salinity stresses were observed in net photosynthesis rate among all 13 purslane accessions. Net photosynthesis rates were decreased with the increasing of salinity levels in all 13 accessions and the highest reduction was recorded at the highest 32 dS m^−1^ salinity compared to control (Figure 2). But interestingly only at 16 dS m^−1^ salinity a slight increase in net photosynthesis rate was found in Ac4, Ac9, and Ac12 compared to control plants (Figure 2). The analysis results showed that the highest reduction (25.95%) in net photosynthesis rate was noted in Ac12 at 32 dS m^−1^ salinity whereas the lowest reduction (0.10%) was found in Ac12 at 24 dS m^−1^ salinity compared to control (Table 4). However, the mean values of all the accessions revealed 3.23%, 4.57%, 7.83%, and 9.96% reductions in net photosynthesis rate, respectively, at 8 dS m^−1^, 16 dS m^−1^, 24 dS m^−1^, and 32 dS m^−1^ salinity, which were statistically significant (*P* < 0.0001, Table 4).

#### 3.2.3. Transpiration Rate

Among all 13 purslane accessions transpiration rate in untreated control plants was greatly significant (*P* < 0.0001) and ranged from 0.33 to 1.32 (mol/m^2^/sec); the highest transpiration rate was recorded in Ac3 and the lowest was recorded in Ac9 (Figure 3). Several purslane accessions among the untreated control plants such as Ac3, Ac5, Ac6, and Ac7 showed nonsignificant similar transpiration rate. Transpiration rate was chronologically reduced due to NaCl-induced salinity stress in most of the purslane accessions with the increasing of salinity levels except in Ac1 and Ac7 at 32 dS m^−1^ salinity and in Ac9 at 8, 16, and 32 dS m^−1^ salinity where increasing of transpiration rate was recorded (Figure 3). The highest reduction (73.48%) in transpiration rate was observed in Ac5 at 24 dS m^−1^ salinity whereas the lowest reduction (9.78%) was found in Ac1 at 8 dS m^−1^ salinity compared to control (Table 5). In contrast, the highest increase (42.15%) in transpiration rate was noted in Ac7 at 32 dS m^−1^ salinity while the lowest increase (3.26%) was found in Ac1 at the same salinity levels in comparison with untreated control plants (Table 5). Nevertheless, on average over all accessions, 26.31%, 35.50%, 47.09%, and 40.96% reductions in transpiration rate were recorded correspondingly at 8 dS m^−1^, 16 dS m^−1^, 24 dS m^−1^, and 32 dS m^−1^ salinity, which were statistically significant (*P* < 0.05, Table 5).

#### 3.2.4. Stomatal Conductance

Stomatal conductance in untreated control 13 purslane accessions varied very significantly (*P* < 0.0001) and ranged from 0.05 to 1.24; the highest value in Ac7 is an ornamental purslane and the lowest value in Ac12 is a common purslane (Table 6). Stomatal conductance in Ac8, Ac9, and Ac12 was recorded as nonsignificant and was statistically similar among all 13 untreated control purslane accessions whereas Ac2, Ac4, Ac5, and Ac13 were also nonsignificantly similar for stomatal conductance (Table 6). Different levels of salinity treatments also significantly (*P* < 0.05) affected the stomatal conductance in purslane plants. The subsequent reductions in stomatal conductance were observed for majority of the accessions with the increasing of salinity levels (Table 6). The highest reduction (97.78%) in stomatal conductance was noted in Ac1 at the highest 32 dS m^−1^ salinity while the lowest reduction (15.38%) was found in Ac2 at 8 dS m^−1^ salinity (Table 6). On the other hand, increases in stomatal conductance were also observed in Ac5 at 8 and 16 dS m^−1^ salinity and in Ac9 at all the salinity levels, respectively. However, the mean stomatal conductance revealed 40.70%, 22.37%, 73.32%, and 56.33% reductions rate, respectively, at 8 dS m^−1^, 16 dS m^−1^, 24 dS m^−1^, and 32 dS m^−1^ salinity, which were statistically significant (*P* < 0.0001, Table 6).

#### 3.2.5. Cluster and Principal Component Analysis (PCA)

In order to assess the patterns of variation UPGMA cluster analysis and PCA were done using biomass yield and physiological parameters where all 13 purslane accessions were grouped into five distinct clusters at 1.19 similarity coefficient level (Figure 4). Among 5 clusters Ac9 was totally separated from others and formed cluster V; Ac5 solely constructed cluster IV; Ac3 was alone in cluster III, whereas cluster II was the largest group that consisted of Ac2, Ac4, Ac6, Ac8, Ac10, Ac12, and Ac13. Cluster I was formed with Ac1 and Ac7. The patterns of cluster analysis were also confirmed by the PCA of three-dimensional (3D) plot which was also the same with the dendrogram (Figure 5). Principal components analysis (PCA) indicated 44% of total variation among all the accessions studied (data not shown).

### 3.3. Effect of Salinity on Stem and Root Histology of Purslane

Electron microscopy observation of the transverse section of stems induced by different salinity levels revealed significant changes in anatomical structures. The most affected parts were cortical tissues (C) compared to other sections. The cell damage may result from stem cortex cell collapse due to salt stress. Stem cortical cells of all the 13 purslane accessions were affected at moderate to the highest salinity stress (16 dS m^−1^, 24 dS m^−1^, and 32 dS m^−1^), whereas root cortical tissues were not affected by augmented salinity levels in case of all the accessions except Ac13. Meanwhile, stem cortical cells of Ac5, Ac9, and Ac12 did not show cell collapse with 0 and 8 dS m^−1^ salinity treatments but later with the increased salinity stress the cortical cell collapse was also increased and the severe cell collapse was observed at the highest salinity (32 dS m^−1^) stress (Figures 6, 7, and 8). More or less the similar results have also been observed in case of stem histology of all other purslane accessions (figure not shown). The root transverse section of Ac4, Ac5, Ac7, and Ac10 did not show any detrimental changes or cell collapse in the cortical tissues at all the salinity levels from 0 dS m^−1^ to 32 dS m^−1^ (Figures 9 and 10) but a slight enlargement of the cortical cells was observed in Ac12 at 32 dS m^−1^ salinity (Figure 11), whereas the same incident was found in Ac13 at the salinity treatments 16 dS m^−1^, 24 dS m^−1^, and 32 dS m^−1^ (Figure 12).

## 4. Discussion

Total biomass yield, that is, fresh weight and dry weight, and physiological characteristics, that is, total chlorophyll content, net photosynthesis rate, transpiration rate, stomatal conductance, water vapor deficit, and stem-root histology, in 13 untreated and salt treated purslane accessions were investigated in this study.

The results showed that untreated control plants greatly varied in the above-mentioned parameters of biomass yield, physiological traits, and stem-root histology. Salt treatment also significantly influenced all parameters investigated in this study. Responses of the 13 purslane accessions to salt treatment were very different from each other and did not follow any particular trend, indicating vast diversity among the purslane accessions collected from different locations in Western Peninsular Malaysia.

Purslane is a very succulent plant containing water about 90% or above both in leaves and in stems. So, the fresh weight of purslane was comparatively higher than dry weight. The elevated salinity stress caused a very high significant reduction in fresh weight of purslane and the fresh weight reduction consecutively increased with the increasing of salinity augmentation. In contrast some of the accessions also achieved significant increase in fresh weight of purslane after salinity application. The highest reduction of fresh weight was observed in Ac8 at all the 4 salinity levels at 8 dS m^−1^ (36.43%), at 16 dS m^−1^ (42.1%), at 24 dS m^−1^ (47.13%), and at 32 dS m^−1^ (54.1%) salinity, respectively, compared to control as well as other accessions (Table 1), whereas in Ac1 salinity-induced increase (2.8%) in fresh weight was seen only at 8 dS m^−1^ and in Ac13 at 8 and 16 dS m^−1^ salinity 9.5% and 15.6% increase in fresh weight were recorded compared to control (Table 1). On the other hand, increase in fresh weight in Ac9 was the highest (23.9%, about 2-fold higher from the lowest to the highest) at 24 dS m^−1^ salinity but with further increasing of salinity at 32 dS m^−1^ the increasing rate was decreased to 16.5% compared to control (Table 1). Salinity-induced fresh weight reduction is a common phenomenon for most of the cultivated crop plants and trees. Behzadifar et al. [26] have described the very high significant reduction of fresh weight of* Catharanthus roseus *at 8 dS m^−1^ salinity. The reductions of fresh weight due to salinity stress have also been investigated by several scientists in several crops in tomato [27] and in* Ocimum basilcum* [28], whereas the increase in fresh weight in* Pennisetum alopecuroides* at 100 mM salinity has been reported by Mane et al. [29]. The reduction in biomass increased with the increase in salinity which is obvious because of disturbances in physiological and biochemical activities under saline conditions as shown by Craine [30] that may be due to the reduction in leaf area and number of leaves [31].

Plants dry matter content is a functional parameter used to assess the plant strategy for resource acquisition and use [32]. NaCl-induced salinity significantly highly affected the total dry matter production in all 13 purslane accessions. The dry matter production in purslane was very low compared to fresh weight due to very high content of water in leaves and stems. The highest significant reduction in dry matter content was recorded in Ac6 at 32 dS m^−1^ salinity which was about 5-fold reduction from the lowest dry matter reduction recorded in Ac5 at the same salinity level (Table 2). But only in case of Ac9 a successive increase in dry matter content was noted from 16 dS m^−1^ up to 32 dS m^−1^ salinity where the highest increase (54.2%) was at 24 dS m^−1^ salinity but later the increasing rate of dry matter content was decreased with the increasing of salinity compared to control (Table 2). The significant decrease in dry matter content of sugar beet cultivars has been described by Dadkhah and Grrifiths [33] at 350 mM salinity stress, whereas at 250 mM salinity the shoot and root dry matter contents were marked decreased in hybrid maize varieties [34] and the increase in dry matter content in* Pennisetum alopecuroides* at 100 mM salinity has also been reported by Mane et al. [35]. Such stimulation in dry matter production under the influence of salinity might be due to the accumulation of inorganic ions and organic solutes for osmotic adaptation while a decrease in dry matter content at the highest salinity levels might be due to the inhibition in hydrolysis of reserved foods and their translocation to the growing shoots [36].

Chlorophyll is the main color agent responsible for photosynthesis. Under adverse circumstances, the chlorophyll level is a good indicator of the photosynthesis function [36]. In our study aggravated salinity stress caused significant changes in chlorophyll content (SPAD value) in all 13 purslane accessions. In most of the cases chlorophyll content was significantly decreased with the increasing of salinity levels. Due to the distinct variation among all 13 purslane accessions their responses to different salinity regimes for chlorophyll content were also different. Reduction of chlorophyll content due to salinity stress is very common in salt-sensitive plant species because of salt toxicity which mostly causes burning of leaves or other succulent parts and degradation of other pigments too. But those are saline tolerant species that can protect themselves from such deterioration of salinity stress. However, it has been found that the chlorophyll level of trees decreases with aggravated salt stress due to enzymatic chlorophyll degradation [37]. The reductions of chlorophyll content in* Catharanthus roseus* [38] and in walnut [39] have been reported due to salinity stress, whereas salinity stressed significant increase in chlorophyll content has also been reported by Nazarbeygi et al. [40] in Canola.

Photosynthesis is the process by which green plants and certain other organisms use the energy of light to convert carbon dioxide and water into the simple sugar glucose. In doing so, photosynthesis provides the basic energy source for virtually all organisms. But the process of photosynthesis is a primary target of many forms of environmental stress, including salinity [41]. In our study we also found both positive and negative effects of salinity on photosynthesis rate of purslane accessions. A great significant decrease in photosynthetic rate was observed in both of the highest salinity levels (24 and 32 dS m^−1^ salinity), whereas only in 3 purslane accessions (Ac4, Ac9, and Ac12) a significant increase in photosynthetic rate was also recorded at the moderate (16 dS m^−1^) salinity stress compared to control (Table 4 and Figure 2). Among all 13 purslane accessions Ac13 was badly affected through all the salinity levels and the highest decrease (25.95%, about 2.5-fold reduction from the lowest to the highest) in photosynthetic rate was noted at 32 dS m^−1^ salinity followed by 22.43% (about 2-fold reduction from the lowest to the highest) at 24 dS m^−1^ salinity and 21.2% (about 2-fold reduction from the lowest to the highest) at 16 dS m^−1^ salinity, respectively, compared to control (Table 4). In contrast the highest increase (7.6%) in photosynthetic rate was observed in Ac12 at 16 dS m^−1^ salinity which was about 2-fold increase compared to the increase observed in Ac4 (4.43%) and Ac9 (4.06%) at the same salinity level compared to control (Table 4). Munns et al. [42] reported photosynthesis and plant growth among the primary processes affected by drought and salinity. Water stress and salinity can affect photosynthesis directly or indirectly by decreasing CO_2_ availability caused by diffusion limitations [43]. Furthermore, Stoeva and Kaymakanova [44] opined that reduced photosynthesis under salinity is attributed not only to stomata closure leading to a reduction of intercellular CO_2_ concentration but also to nonstomata factors.

Transpiration performs a significant physiological role in maintaining the osmotic concentration in the plant. If the osmotic concentration is higher or lower than the normal levels, the physiological process of the plants will be disrupted. Exposure of plants to salt stress results in changes in most physiological and biochemical processes resulting in a disturbance of normal growth and development [45]. Aggravated salinity stress caused a great significant reduction that is transpiration rate in all 13 purslane accessions and the rate of reductions was increased with the increasing of salinity levels with an exceptional increasing in Ac1 (3.26%) at 32 dS m^−1^ salinity, 42.15% increasing in Ac7 at 32 dS m^−1^ salinity, 27.3% increase at 8 dS m^−1^ salinity, and 12.12% increase at 16 dS m^−1^ salinity, and 36.7% increase was recorded at 32 dS m^−1^ salinity, respectively, in Ac9 compared to control (Table 5). On the other hand, the highest reduction was seen in Ac5 which was about 2-fold greater from the lowest value at 24 dS m^−1^ salinity in Ac1 compared to control, whereas the second lowest reduction of transpiration even at the highest salinity stress was recorded in Ac13 meaning that this accession was more capable of surviving against salinity compared to other affected accessions. Hatamnia et al. [46] have concluded the decreased transpiration rate due to 200 mM salinity stress in tobacco cultivars. NaCl stress-induced remarkable reduction in transpiration in mustard has also been reported by Jamil and Rha [47].

Stomata are the pores on a leaf surface through which plants regulate the uptake of carbon dioxide (CO_2_) for photosynthesis against the loss of water via transpiration. The stomatal control responses of plants are influenced by several biotic and abiotic factors including drought and salinity. All through our study stomatal conductance was very significantly affected by different levels of salinity stresses. Stomatal conductance greatly decreased with the increasing of salinity levels in all 13 purslane accessions except Ac5 at 8 and 16 dS m^−1^ salinity and in Ac9 at all salinity levels where a significant increase was found compared to control. Considering the salinity level-wise reduction of stomatal conductance at 24 dS m^−1^ salinity similar stomatal conductance was observed in Ac3, Ac4, Ac8, Ac10, Ac11, Ac12, and Ac13, respectively, compared to control, whereas at 32 dS m^−1^ salinity similar response was also noted in Ac1, Ac2, Ac3, Ac4, Ac5, Ac6, and Ac8, respectively, as well as Ac10, Ac11, Ac12, and Ac13 (Table 6). Moradi and Ismail [48] postulated that photosynthesis is inhibited in the presence of salinity through either reduction in stomatal conductance or such nonstomatal factors as a reduction in chlorophyll pigments to absorb enough light. Furthermore, the reduction of stomatal conductance and mesophyll might contribute to the inhibition of photosynthesis under salt stress [49].

Cluster analysis is a multivariate technique that can group individuals or objects on the basis of their characteristics. Individuals having similar descriptions are mathematically congregated into the same cluster [50]. Distance, similarity, and relatedness of varieties are the foundation of this method. The UPGMA constructed dendrogram revealed 5 clusters where Ac9 was mostly different from all others proving the highest salt-tolerant accession compared to others and possesses the highest diversity compared to Ac2 and Ac11. For new improved variety development the most judicious crossing combination can be made with Ac9 and Ac2 or Ac11 or Ac6 or Ac8 that will bring about the greater genetic diversity [51].

The stem histology of purslane especially cortical tissues was very badly affected by different levels of salinity stress compared to control, whereas no significant variation was seen in root histology of purslane at any salinity levels except Ac12 at the highest 32 dS m^−1^ salinity and Ac13 at 16, 24, and 32 dS m^−1^ salinity where a slight enlargement of the cortical cells was observed (Figures 11 and 12). Rewald et al. [52] reported that plants roots are potentially the first sites of damage or line of defense due to the direct contact with soil solution and the first to encounter excess salinity. On the other hand, being the outermost cell layers after the epidermis/exodermis, the cortex is the first tissue to encounter salinity. Very recently, Boughalleb et al. [53] found that the root cortex thickness was promoted under 100–200 mM NaCl in the xerohalophyte shrubs* Nitraria retusa *and* Atriplex halimus. *However, in some cases, salinity imposed a reduction in cortex development. Akram et al. [54] reported a decreased size of the cortex under salinity stress in three varieties of* Triticum aestivum*; the most salt-sensitive variety showed a more pronounced decrease. Similarly, the cortical parenchyma in* Chloris gayana *decreased under saline conditions [55], and reductions of cortex thickness under high salinity were also reported in shrubs [53] and tree roots [56]. Hakim et al. [57] conducted an experiment on rice and opined that cortical cells of MR211 and MR232 did not show cell collapse up to 8 dS m^−1^ salinity levels compared to susceptible checks (IR20 and BRRI dhan29). The significant damage of cortical tissues in salt-sensitive turfgrass species has also been reported by Uddin et al. [58].

## 5. Conclusions

Global warming and industrialization are directly related to environmental changes, sea level rising and severe soil and water salinity, resulting in unsuitable existence for many important crop species. Considering this urgency, in our study we have tested 13 collected purslane accessions for biomass yield loss and physiological and stem-root anatomical characteristics on augmented salinity stress. Analysis results revealed that though there had been significant variation among all 13 purslane accessions for measured parameters commonly it has been proved as a high salt-tolerant crop plant capable of producing satisfactory amount of dry matter content which is a great demand for any salt-tolerant plant species. All through the experiment accession-wise complex results were found. Different accessions showed different performance in varied salinity stress. But one common trend was more or less that all accessions were affected at the highest salinity compared to control as well as moderate to lower salinity. Considering salinity effect on purslane physiology, increase in chlorophyll content was seen in Ac2, Ac4, Ac6, and Ac8 at 16 dS m^−1^ salinity, whereas, Ac4, Ac9, and Ac12 showed increased photosynthesis at the same salinity levels compared to control. Anatomically, stem cortical tissues of Ac5, Ac9, and Ac12 were unaffected at control and 8 dS m^−1^ salinity but root cortical tissues did not show any significant damage except a bit enlargement in Ac12 and Ac13. Overall, salinity stressed among all 13 purslane accessions considering biomass production, physiological growth, and anatomical development Ac9 was the best salt-tolerant purslane accession which produced the highest amount of fresh and dry weight and Ac13 was the most affected accession. It was also found that the ornamental purslane showed more salt tolerance than common purslane. We hope our findings will benefit readers, consumers, and producers to cultivate purslane vegetables in any type of soils especially salinity affected areas.

## Figures and Tables

**Figure 1:** Effect of salinity on total chlorophyll content of 13 purslane accessions. Each bar represents mean values (±SE) of three replicates. Mean values with different lower case letters within a group (i.e., accessions) are significantly different at *P* < 0.05.

**Figure 2:** Effect of salinity on net photosynthesis rate of 13 purslane accessions. Each bar represents mean values (±SE) of three replicates. Mean values with different lower case letters within a group (i.e., accessions) are significantly different at *P* < 0.05.

**Figure 3:** Effect of salinity on transpiration rate of 13 purslane accessions. Each bar represents mean values (±SE) of three replicates. Mean values with different lower case letters within a group (i.e., accessions) are significantly different at *P* < 0.05.

**Figure 4:** A UPGMA dendrogram of measured traits derived from 13 salinity tolerant purslane accessions.

**Figure 5:** A three-dimensional PCA plot indicating variations among 13 salinity tolerant purslane accessions.

**Figure 6:** Scanning electron micrographs showing salinity effects on purslane stem histology of Ac5.

**Figure 7:** Scanning electron micrographs showing salinity effects on purslane stem histology of Ac9.

**Figure 8:** Scanning electron micrographs showing salinity effects on purslane stem histology of Ac12.

**Figure 9:** Scanning electron micrographs showing salinity effects on purslane root histology of Ac4.

**Figure 10:** Scanning electron micrographs showing salinity effects on purslane root histology of Ac10.

**Figure 11:** Scanning electron micrographs showing salinity effects on purslane root histology of Ac12.

**Figure 12:** Scanning electron micrographs showing salinity effects on purslane root histology of Ac13.

**Table 1:** Effect of salinity on fresh weight of 13 purslane accessions.

Purslane accessions	Fresh weight (g)				
	Salinity level (dS m^−1^)				
	0	8	16	24	32
Ac1	225.0 ± 1.28 e	231.33 ± 4.44 b (+2.81)	203.78 ± 3.39 b (9.43)	192.49 ± 2.62 b (14.45)	187.37 ± 1.13 b (16.72)
Ac2	213.58 ± 1.72 f	203.14 ± 3.45 e (4.88)	193.58 ± 2.70 c (9.36)	188.93 ± 2.33 bc (11.54)	171.58 ± 1.67 d (19.66)
Ac3	190.50 ± 1.83 g	188.79 ± 1.86 f (0.89)	177.93 ± 2.62 d (6.59)	181.37 ± 1.92 bc (4.79)	177.68 ± 1.86 c (6.73)
Ac4	187.0 ± 3.24 g	149.16 ± 2.23 g (20.24)	112.32 ± 1.83 g (39.94)	117.30 ± 1.93 g (37.27)	106.31 ± 1.35 h (43.15)
Ac5	134.16 ± 1.24 i	121.31 ± 1.78 h (9.58)	129.48 ± 1.66 e (3.39)	131.28 ± 1.91 f (2.15)	113.58 ± 1.65 g (15.34)
Ac6	279.0 ± 2.71 c	229.0 ± 2.82 b (17.92)	174.72 ± 1.59 d (37.38)	154.68 ± 11.28 e (44.56)	159.87 ± 2.44 e (42.69)
Ac7	230.0 ± 3.67 e	223.51 ± 1.67 c (2.82)	174.97 ± 2.14 d (23.93)	168.94 ± 2.29 d (26.55)	151.60 ± 2.77 f (34.09)
Ac8	341.03 ± 2.39 a	216.82 ± 2.37 d (36.42)	197.43 ± 3.76 bc (42.11)	180.29 ± 2.82 cd (47.13)	156.61 ± 2.68 ef (54.08)
Ac9	305.17 ± 2.02 b	248.61 ± 2.68 a (18.53)	346.97 ± 2.15 a (+13.69)	378.15 ± 3.22 a (+23.91)	355.68 ± 1.81 a (+16.55)
Ac10	149.17 ± 1.28 h	114.53 ± 1.64 i (23.22)	103.43 ± 1.74 h (30.66)	98.26 ± 2.39 h (34.13)	89.30 ± 1.91 j (40.14)
Ac11	242.0 ± 1.66 d	185.0 ± 2.43 f (23.55)	174.83 ± 2.28 d (27.76)	169.56 ± 1.67 d (29.93)	161.79 ± 2.50 e (33.14)
Ac12	129.48 ± 1.73 i	112.94 ± 1.37 i (12.77)	105.14 ± 1.95 h (18.79)	93.40 ± 1.38 h (27.27)	86.98 ± 2.31 j (32.82)
Ac13	103.66 ± 3.79 j	113.52 ± 1.82 i (+9.51)	119.81 ± 1.22 f (+15.58)	101.30 ± 2.81 h (2.78)	99.11 ± 3.32 i (4.39)

Mean	209.98 ± 71.18 a	179.82 ± 51.01 b (14.36)	170.34 ± 64.57 c (18.88)	165.84 ± 73.28 d (21.02)	155.19 ± 69.73 e (26.09)

Values and ±SE with different lower case letters in a row are significantly different at *P* < 0.05. Values in the parentheses indicate percent compared to the untreated control (0 dS m^−1^) plants. Plus (+) symbol indicates % increase in fresh weight compared to control.

**Table 2:** Effect of salinity on dry matter contents of 13 purslane accessions.

Purslane accessions	Dry weight (g)				
	Salinity level (dS m^−1^)				
	0	8	16	24	32
Ac1	16.27 ± 1.37 bc	17.13 ± 1.80 bc (+5.29)	13.10 ± 1.23 bc (13.1)	9.23 ± 1.33 e–g (9.23)	8.33 ± 1.12 ef (8.33)
Ac2	15.39 ± 1.74 bc	13.58 ± 1.60 d (11.76)	10.34 ± 0.84 d (10.34)	9.18 ± 0.94 e–g (9.18)	8.42 ± 1.75 d–f (8.42)
Ac3	23.55 ± 1.86 a	21.39 ± 1.79 a (21.39)	19.29 ± 2.01 a (19.29)	20.16 ± 1.27 b (20.16)	18.51 ± 0.65 b (18.51)
Ac4	15.55 ± 0.66 bc	13.97 ± 2.11 cd (13.97)	10.70 ± 0.83 d (10.7)	8.95 ± 0.47 e–g (8.95)	8.66 ± 0.47 d–f (8.66)
Ac5	7.94 ± 0.19 d	6.45 ± 0.86 f (6.45)	6.74 ± 0.51 f (6.74)	7.81 ± 0.42 fg (7.81)	5.39 ± 0.41 g (5.39)
Ac6	20.67 ± 0.41 ab	17.77 ± 0.29 ab (17.77)	10.02 ± 0.15 d (10.02)	14.38 ± 0.43 c (14.38)	7.55 ± 0.30 e–g (7.55)
Ac7	15.91 ± 0.32 bc	13.24 ± 0.41 d (13.24)	14.17 ± 0.32 b (14.17)	12.77 ± 0.36 cd (12.77)	12.04 ± 0.25 c (12.04)
Ac8	16.63 ± 6.94 bc	11.57 ± 0.28 de (11.57)	11.16 ± 0.33 cd (11.16)	10.92 ± 0.34 de (10.92)	9.98 ± 0.17 c–e (9.98)
Ac9	15.50 ± 0.37 bc	13.48 ± 0.37 d (13.48)	21.30 ± 0.47 a (21.3)	23.90 ± 0.37 a (23.9)	23.40 ± 0.29 a (23.4)
Ac10	10.10 ± 0.19 cd	8.60 ± 0.21 ef (8.6)	7.44 ± 0.31 ef (7.44)	7.13 ± 0.22 g (7.13)	6.89 ± 0.29 fg (6.89)
Ac11	18.84 ± 2.33 ab	14.0 ± 1.61 cd (14.0)	13.43 ± 1.74 bc (13.43)	12.47 ± 0.66 cd (12.47)	11.08 ± 2.10 cd (11.08)
Ac12	11.99 ± 0.18 cd	14.41 ± 0.28 b–d (14.41)	9.46 ± 0.15 de (9.46)	7.72 ± 0.36 fg (7.72)	6.33 ± 0.48 fg (6.33)
Ac13	12.05 ± 0.20 cd	12.27 ± 0.88 d (12.27)	11.34 ± 0.76 cd (11.34)	9.58 ± 0.92 ef (9.58)	7.93 ± 0.31 e–g (7.93)

Mean	15.41 ± 4.23 a	13.68 ± 3.80 b (11.24)	12.19 ± 4.19 c (20.91)	11.86 ± 5.05 d (23.05)	10.35 ± 5.14 e (32.88)

Mean values ± SE with different lower case letters in a row are significantly different at *P* < 0.0001. Values in the parentheses indicate percent compared to the untreated control (0 dS m^−1^) plants. Plus (+) symbol indicates % increase in fresh weight compared to control.

**Table 3:** Effect of salinity on total chlorophyll content (% reduction) of 13 purslane accessions.

Accession number	Total chlorophyll contents (SPAD value) (% changes)			
	8 dS m^−1^	16 dS m^−1^	24 dS m^−1^	32 dS m^−1^
Ac1	4.78	3.98	4.78	3.98
Ac2	+1.87	+2.62	11.99	12.36
Ac3	15.02	9.01	9.61	6.31
Ac4	5.39	+3.29	12.57	21.86
Ac5	14.29	11.11	17.06	21.43
Ac6	2.36	+3.37	9.09	19.19
Ac7	17.08	18.63	21.12	39.44
Ac8	+3.64	+1.82	11.21	18.79
Ac9	11.38	13.01	23.59	25.14
Ac10	5.20	6.65	8.38	12.43
Ac11	0.32	3.90	16.88	18.83
Ac12	7.54	21.51	21.23	34.36
Ac13	4.51	4.23	5.07	16.34

Mean	6.45	6.55	13.51	19.72

The plus symbol (+) indicates % increase of chlorophyll contents.

**Table 4:** Effect of salinity on net photosynthesis rate of 13 purslane accessions.

Accession number	Net photosynthesis (*μ*mol CO_2_/m^2^/sec) (% changes)			
	8 dS m^−1^	16 dS m^−1^	24 dS m^−1^	32 dS m^−1^
Ac1	7.83	13.50	17.32	16.85
Ac2	5.20	11.26	13.37	16.60
Ac3	1.28	2.51	3.56	8.09
Ac4	1.56	+4.43	3.12	4.93
Ac5	2.06	3.98	4.89	7.18
Ac6	1.38	3.32	5.27	6.85
Ac7	1.04	5.25	7.13	9.71
Ac8	1.37	2.59	6.55	9.48
Ac9	3.35	+4.06	0.81	1.22
Ac10	2.10	6.36	7.68	8.87
Ac11	0.82	3.20	7.86	8.82
Ac12	2.60	+7.60	0.10	3.03
Ac13	10.78	21.20	22.43	25.95

Mean	3.23	4.57	7.83	9.96

The plus symbol (+) indicates % increase of net photosynthesis rate.

**Table 5:** Effect of salinity on transpiration rate of 13 purslane accessions.

Accession number	Transpiration rate (% reduction and increase)			
	8 dS m^−1^	16 dS m^−1^	24 dS m^−1^	32 dS m^−1^
Ac1	9.78	26.09	47.83	+3.26
Ac2	25.23	40.54	50.45	63.06
Ac3	41.67	30.30	50.76	72.73
Ac4	19.09	30.91	20.91	67.27
Ac5	34.09	53.03	73.48	34.09
Ac6	41.46	32.52	44.72	64.23
Ac7	32.23	43.80	50.41	+42.15
Ac8	22.22	43.52	47.22	63.89
Ac9	+27.27	+12.12	27.27	+36.36
Ac10	21.62	38.74	48.65	64.86
Ac11	20.72	31.53	38.74	48.65
Ac12	30.67	36.00	49.33	58.67
Ac13	24.05	26.58	41.77	13.92

Mean	26.31	35.50	47.09	40.96

The plus symbol (+) indicates % increase of transpiration rate.

**Table 6:** Effect of salinity on stomatal conductance of 13 purslane accessions.

Purslane accessions	Stomatal conductance (cm/sec)				
	Salinity level (dS m^−1^)				
	0	8	16	24	32
Ac1	0.91 ± 0.03 b	0.42 ± 0.02 b (53.33)	0.22 ± 0.02 bc (75.56)	0.05 ± 0.02 b (94.44)	0.02 ± 0.01 c (97.78)
Ac2	0.13 ± 0.01 d	0.11 ± 0.03 de (15.38)	0.09 ± 0.02 c (30.77)	0.05 ± 0.01 b (61.54)	0.03 ± 0.01 c (76.92)
Ac3	0.31 ± 0.02 c	0.18 ± 0.05 cd (41.94)	0.07 ± 0.03 c (77.42)	0.04 ± 0.01 b (87.10)	0.03 ± 0.01 c (90.32)
Ac4	0.12 ± 0.01 d	0.09 ± 0.01 de (25.0)	0.06 ± 0.01 c (50.0)	0.04 ± 0.01 b (66.67)	0.02 ± 0.01 c (83.33)
Ac5	0.10 ± 0.01 d	0.11 ± 0.01 de (+10.0)	0.59 ± 0.44 b (+490.0)	0.05 ± 0.02 b (50.0)	0.05 ± 0.01 c (50.0)
Ac6	0.16 ± 0.03 cd	0.07 ± 0.01 de (56.25)	0.08 ± 0.01 c (50.0)	0.07 ± 0.01 b (56.25)	0.04 ± 0.01 c (75.0)
Ac7	1.24 ± 0.20 a	0.26 ± 0.04 c (79.05)	0.13 ± 0.02 bc (89.52)	0.08 ± 0.01 b (93.55)	0.47 ± 0.04 b (62.10)
Ac8	0.09 ± 0.01 d	0.03 ± 0.02 e (66.67)	0.03 ± 0.01 c (66.67)	0.02 ± 0.01 b (77.78)	0.03 ± 0.01 c (66.67)
Ac9	0.06 ± 0.01 d	0.69 ± 0.14 a (+1050.0)	1.46 ± 0.38 a (+2333.0)	0.49 ± 0.20 a (+716.67)	0.87 ± 0.45 a (+1350.0)
Ac10	0.22 ± 0.01 cd	0.08 ± 0.02 de (63.64)	0.05 ± 0.02 c (77.27)	0.02 ± 0.01 b (90.91)	0.01 ± 0.01 c (95.45)
Ac11	0.21 ± 0.02 cd	0.06 ± 0.01 de (71.43)	0.04 ± 0.01 c (80.95)	0.03 ± 0.03 b (85.71)	0.01 ± 0.01 c (95.24)
Ac12	0.05 ± 0.01d	0.04 ± 0.01 e (20.0)	0.02 ± 0.01 c (60.0)	0.02 ± 0.01 b (60.0)	0.02 ± 0.04 c (60.0)
Ac13	0.12 ± 0.01 d	0.06 ± 0.01 de (50.00)	0.04 ± 0.01 c (66.67)	0.03 ± 0.01 b (75.0)	0.02 ± 0.01 c (83.33)

Mean	0.29 ± 0.36 a	0.17 ± 0.19 c (40.70)	0.22 ± 0.4 b (22.37)	0.08 ± 0.13 e (73.32)	0.12 ± 0.26 d (56.33)

Mean values and ±SE with different lower case letters in a row are significantly different at *P* < 0.05. Values in the parentheses indicate percent compared to the untreated control (0 dS m^−1^) plants. The minus symbol (−) indicate % increase of transpiration rate.
